The article "Correlation between Changes in Serum RBP4, hs-CRP, and IL-27 Levels and Rosuvastatin in the Treatment of Coronary Heart Disease" was published in 2021. Journal: J Healthc Eng.

# Correlation between Changes in Serum RBP4, hs-CRP, and IL-27 Levels and Rosuvastatin in the Treatment of Coronary Heart Disease

**DOI:** 10.1155/2021/8476592

**Published:** 2021-12-15

**Authors:** Yali Wang, Changrui Zhou, Tianlian Yu, Feng Zhao

**Affiliations:** ^1^Department of Internal Medicine-Cardiovascular, Dongying Traditional Chinese Medicine Hospital, Dongying 257055, Shandong Province, China; ^2^Department of Clinical Laboratory, Dongying Traditional Chinese Medicine Hospital, Dongying 257055, Shandong Province, China

## Abstract

**Objective:**

To investigate the correlation between changes in serum RBP4, hs-CRP, and IL-27 levels and rosuvastatin in the treatment of coronary heart disease (CHD).

**Methods:**

One hundred and twenty patients with CHD admitted in our hospital were selected as the research object, including 60 patients with acute coronary syndrome as the ACS group, and 60 patients with stable angina as the SA group. Another 60 patients without CHD who were examined in our hospital at the same time were included in the non-CHD group. The patients with CHD were further divided into the control group (CG) (*n* = 42, with routine treatment) and the study group (SG) (*n* = 78, with routine treatment and rosuvastatin) to measure serum RBP4, hs-CRP, and IL-27 levels and analyze the correlation between each index and rosuvastatin in the treatment of CHD.

**Results:**

After retrospective analysis, no significant difference was found among the ACS group, the SA group, and the non-CHD group (*P* > 0.05). As for serum RBP4, hs-CRP, and IL-27 levels, ACS group > SA group > non-CHD group, with obvious differences among groups (*P* < 0.05). After Spearman correlation analysis, a positive correlation was observed between Gensini score and serum RBP4, hs-CRP, and IL-27 levels in patients with CHD (*P* < 0.05). After treatment, serum RBP4, hs-CRP, and IL-27 levels were gradually reduced. At 4 weeks after treatment, serum RBP4, hs-CRP, and IL-27 levels of the CG and the SG were decreased conspicuously, and compared with the control, each index of the SG was obviously lower (*P* < 0.05).

**Conclusion:**

Serum RBP4, hs-CRP, and IL-27 play an important role in the occurrence and development of CHD, with a positive correlation to the Gensini score, which can indicate the severity of cardiovascular disease to a certain extent. Meanwhile, rosuvastatin can remarkably reduce serum RBP4, hs-CRP, and IL-27 levels, which is of significance for prognosis.

## 1. Introduction

Coronary heart disease (CHD) is a kind of atherosclerotic heart disease, with some triggering factors such as age, gender, and family history, and other changeable factors including hypertension, hyperglycemia, dyslipidemia, and bad lifestyle (excessive drinking and smoking, imbalanced diet, etc.) [1–4]. A large number of clinical studies have shown that inflammatory response plays an important role in changing coronary plaques, and many inflammatory factors can predict the risk of CHD [5–8]. The study of Farrokhian et al. [9] have pointed out that high-sensitivity C-reactive protein (hs-CRP) and interleukin-27 (IL-27) are all involved in the body's inflammatory response, which can reflect the degree of inflammation of patients. In addition, retinol binding protein (RBP4) also shows high expression in patients with CHD, and it is often combined with high levels of other inflammatory factors. At present, there are few reports on the correlation between the changes of serum RBP4, hs-CRP, and IL-27, and CHD. According to the author's clinical experience, drug treatment is always the basis of controlling CHD. Moreover, the results of a clinical endpoint published by American Heart Association in 2005 [10] confirmed that low LDL cholesterol levels will be more beneficial for patients with CHD, so lipid lowering is especially emphasized in clinical practice. The new statins-related drug, rosuvastatin, mainly acts on the liver (the cholesterol lowering target organ), which is faster and stronger in lipid lowering than other drugs, and CHD is caused by the formation of a plaque in the inner wall of the coronary vasculature that undergoes stiffening, and therefore lipids are closely related to plaque growth as they are basically the raw material of atherosclerotic plaques. Hence, it is of great clinical value to study rosuvastatin in the treatment of CHD because of its ability to inhibit plaque growth. In this respect, rosuvastatin is more effective than other statins. Therefore, rosuvastatin was used as an intervention factor to observe the changes of serum RBP4, hs-CRP, and IL-27 levels in patients with CHD after rosuvastatin treatment, so as to analyze the correlation and provide a new medical basis for disease control.

## 2. Methods

### 2.1. Screening and Grouping

One hundred and twenty patients with CHD admitted in our hospital were selected as the research object, including 60 patients with acute coronary syndrome as the ACS group, and 60 patients with stable angina as the SA group. Another 60 patients without CHD who examined in our hospital at the same time were included into the non-CHD group. The patients with CHD were further divided into the control group (CG) (*n* = 42, with routine treatment) and the study group (SG) (*n* = 78, with routine treatment and rosuvastatin). The study was approved by the Hospital Ethnic Community.

### 2.2. Inclusion Criteria

All patients with acute coronary syndrome met the relevant diagnostic criteria in the guidelines for the diagnosis and treatment of acute ST-segment elevation myocardial infarction (2015) [11] and the guidelines for the diagnosis and treatment of non-ST-segment elevation acute coronary syndrome (2016) [12]. Patients with stable angina pectoris met the diagnostic criteria in the guidelines for the diagnosis and treatment of chronic stable angina pectoris [13], and selective coronary angiography showed that the coronary artery stenosis was more than 50% in single or multiple branches. (2) The clinical data of the patients were complete. (3) No acute infectious lesion was found by blood routine examination. (4) Patients and their family members understood the study and signed the consent form.

### 2.3. Exclusion Criteria

(1) Patients had transient cerebral ischemia or stroke recently. (2) Patients were complicated with autoimmune diseases, other severe organic diseases, and malignant tumors. (3) Patients had a history of hyperthyroidism or hypothyroidism. (4) Patients were without good control of underlying diseases (hypertension, diabetes mellitus, and hyperlipidemia) or had unstable conditions. (4) Patients had cognitive disorder and communication disorder. (6) Patients had low treatment compliance or quit the trial in the middle of treatment.

### 2.4. Methods

#### 2.4.1. Treatment Methods

The changes of electrocardiogram, blood pressure, heart rate, respiration, blood oxygen saturation, and cardiac function were closely monitored to take timely treatment measures. Patients with low blood oxygen saturation were given continuous oxygen inhalation [14]. Drug therapy was conducted for antithrombus (antiplatelet and anticoagulation), alleviating angina pectoris (nitrates), reducing myocardial oxygen consumption (beta receptor blocker), and adjusting lipid to stabilize plaques (statins drugs) [15]. Patients in the SG were treated with rosuvastatin on the basis of routine treatment (Specification: 10 mg; Manufacturer: Pfizer Pharmaceutical Co., Ltd.; NMPA Approval No. H20051408), with the dosage of 10 mg/day and the maximum dose of 30 mg/day, which could be taken once at any time and was not limited by meal time.

#### 2.4.2. Observation Indexes

After admission, 5 ml of fasting venous blood of patients was taken in the morning, and centrifuged at 3000 r/min for 10 minutes to take the upper serum, which was stored at −80 °C for testing. Serum RBP4, hs-CRP, and IL-27 levels were measured by enzyme-linked immunosorbent assay (ELISA). The kit was from Shanghai Kamaishu Biological Technology Co., Ltd. The specific operation was performed in strict accordance with the specification on the kits.

#### 2.4.3. Gensini Score

The degree of lesion was evaluated by the coronary stenosis score (Gensini score), which included the coronary stenosis degree score and lesion site score [16]. (1) Stenosis degree score: the stenosis degree under 25% was recorded as 1 point; 25–50% as 2 points; 51–75% as 4 points; 76–90% as 8 points; 91–99% as 16 points; and 100% as 32 points. (2) The lesion site score was the product of a single lesion score and coefficient. ① Left trunk: 5; ② Opening of circumflex artery: 3.5; ③ Proximal segment of circumflex artery: 2.5; ④ Proximal anterior descending branch: 2.5; ⑤ Middle anterior descending branch: 1.5; ⑥ Aorta and first diagonal branch: 1.0; ⑦ Distal segment of circumflex artery: 1; ⑧ Left branches: 0.5; ⑨ Other branches: 1.0. 1–30 points was regarded as mild; 31–60 as moderate; and >60 as severe.

### 2.5. Statistical Processing

All statistical data of the study were processed by SPSS22.0 to calculate the difference between groups, and the pictures were graphed by GraphPad Prism 7 (GraphPad Software, San Diego, USA). The study included enumeration data and measurement data which were expressed as [*n* (%)] and ($\bar{x}$ ± *s*), respectively, and the study used *X*^2^ test and *t*-test. The differences were statistically significant at *P* < 0.05.

## 3. Results

### 3.1. General Data

After retrospective analysis, no significant difference was found among the ACS group, the SA group, and the non-CHD group (*P* > 0.05), see Table 1.

### 3.2. Changes of Serum RBP4, Hs-CRP, and IL-27 Levels

As for serum RBP4, hs-CRP, and IL-27 levels, ACS group > SA group > non-CHD group, with obvious differences among groups (*P* < 0.05); see Table 2.

### 3.3. Correlation between Gensini Score and Serum RBP4, Hs-CRP, and IL-27 Levels

After Spearman correlation analysis, a positive correlation was observed between Gensini score and serum RBP4, hs-CRP, and IL-27 levels in patients with CHD (*P* < 0.05), see Table 3.

### 3.4. Influence of Rosuvastatin on Serum RBP4, Hs-CRP, and IL-27 Levels

One hundred and twenty patients with CHD were further divided into the CG (*n* = 42, with routine treatment) and the SG (*n* = 78, with routine treatment and rosuvastatin). After treatment, serum RBP4, hs-CRP, and IL-27 levels were gradually reduced. At 4 weeks after treatment, serum RBP4, hs-CRP, and IL-27 levels of the CG and the SG were decreased conspicuously, and compared with the control; each index of the SG was obviously lower (*P* < 0.05), see Figures 1–3.

## 4. Discussion

As people's life is changing, CHD has become a threat to human life and health. More and more attention is paid to the important role of local or systemic inflammatory reaction in the occurrence and development of CHD. Hs-CRP and IL-27 are essential inflammatory factors. On the one hand, hs-CRP is an acute phrase response protein, which is mainly produced by the liver. When the body has trauma, inflammation or stress reaction, the liver produces hs-CRP, thus resulting in an increase of serum hs-CRP. Meanwhile, hs-CRP is also a common nonspecific inflammatory factor, which participates in the occurrence and development of atherosclerosis through many different ways according to relevant studies [17–20]. Li et al. [21] found that hs-CRP can trigger vascular endothelial injury by activating the complement system, and coagulation and fibrinolysis imbalance by activating the coagulation system and fibrinolysis system, eventually increasing the risk of cardiovascular diseases. On the other hand, IL-27 is a covalent double-stranded cytokine, which can combine with various immune cells, mediate the immune system, and involve in the coronary atherosclerosis [22]. Recent studies have found that the stability of coronary plaques determines the severity of coronary artery lesions. RBP4 is a newly identified circulating adipokine involved in insulin resistance, which is the vital extracellular transporter responsible for binding and transporting retinol in the blood. Studies have discovered that RBP4 can improve atherosclerosis by influencing the metabolism of lipid and glucose and further changing the stability of coronary plaques [23, 24]. At the same time, the role of serum RBP4, hs-CRP, and IL-27 levels has been proved by related animal experiments in other countries. In this study, as for serum RBP4, hs-CRP, and IL-27 levels, ACS group > SA group > non-CHD group, with obvious differences among groups (*P* < 0.05), which was consistent with the study result of Kotseva et al. [25]. After Spearman correlation analysis, a positive correlation was observed between Gensini score and serum RBP4, hs-CRP, and IL-27 levels in patients with CHD (*P* < 0.05), which further confirmed that serum RBP4, hs-CRP, and IL-27 levels could accurately reflect the severity of CHD. Therefore, RBP4, hs-CRP, and IL-27 were considered as the important observation indexes for the treatment of CHD in this study.

Epidemiological studies have shown that abnormal lipid metabolism mostly leads to the deposition of lipid particles in the intima of the arterial wall, which is also an indispensable pathogenesis of atherosclerosis; while rosuvastatin, a selective HMG-CoA reductase inhibitor, is able to increase the number of hepatic low-density lipoprotein (LDL) receptors on cell surface, promote the absorption and catabolism of LDL, inhibit the hepatic synthesis of LDL, and therefore reduce the total number of very low-density lipoprotein (VLDL) and LDL microparticles. Hence, one hundred and twenty patients with CHD were further divided into the CG (*n* = 42, with routine treatment) and the SG (*n* = 78, with routine treatment and rosuvastatin). After treatment, serum RBP4, hs-CRP, and IL-27 levels were gradually reduced. At 4 weeks after treatment, serum RBP4, hs-CRP, and IL-27 levels of the CG and the SG were decreased conspicuously, and compared with the control; each index of the SG was obviously lower (*P* < 0.05). The results showed that rosuvastatin had obvious anti-inflammatory effect at 4 weeks of treatment on the ground that serum RBP4, hs-CRP, and IL-27 levels were conspicuously reduced, the development of coronary plaques was inhibited, and the stability of the plaques was strengthened. However, compared with the CG, serum RBP4, hs-CRP, and IL-27 levels of the SG were slightly lower, which verified the sensitivity of rosuvastatin for CHD. Therefore, it also provided a theoretical basis for clinical medication that the dosage of rosuvastatin should be increased to control the disease in the first 4 weeks of treatment and then returned to be normal. This retrospective study also has some shortcomings. The specific dosage of rosuvastatin has not been researched. Therefore, further exploration should be carried out to clarify the effects of different doses of rosuvastatin on the serum RBP4, hs-CRP, and IL-27 levels in various stages.

To sum up, serum RBP4, hs-CRP, and IL-27 play an important role in the occurrence and development of CHD, with a positive correlation to the Gensini score, which can indicate the severity of cardiovascular disease to a certain extent. Meanwhile, rosuvastatin can remarkably reduce serum RBP4, hs-CRP, and IL-27 levels, which is of significance for prognosis and improvement of the condition of CHD clinically, and can imply the development and progression of disease more accurately.

## Figures and Tables

**Figure 1:** Comparison of changes of RBP4 level. Note: The abscissa indicated the time nodes, and the ordinate indicated the level, mg/L. The RBP4 levels of the CG before treatment, at 4 weeks, 8 weeks, and 12 weeks of treatment were (35.76 ± 10.42), (26.64 ± 8.41), (24.49 ± 6.11), and (23.06 ± 5.57). The RBP4 levels of the SG before treatment, at 4 weeks, 8 weeks, and 12 weeks of treatment were (35.34 ± 10.35), (23.55 ± 6.87), (22.26 ± 6.15), and (20.92 ± 5.72). ^∗^indicates the obvious difference in the RBP4 level at 4 weeks of treatment between both groups (*t* = 2.170, *P* = 0.032).

**Figure 2:** Comparison of changes of hs-CRP level. Note: The abscissa indicated the time nodes, and the ordinate indicated the level, mg/L. The hs-CRP levels of the CG before treatment, at 4 weeks, 8 weeks, and 12 weeks of treatment were (5.41 ± 2.60), (4.56 ± 1.44), (4.06 ± 1.93), and (3.88 ± 1.60). The hs-CRP levels of the SG before treatment, at 4 weeks, 8 weeks, and 12 weeks of treatment were (5.45 ± 2.63), (3.77 ± 1.12), (3.53 ± 1.05), and (3.41 ± 1.01). ^∗^indicates the obvious difference in the hs-CRP level at 4 weeks of treatment between both groups (*t* = 3.327, *P* = 0.001).

**Figure 3:** Comparison of changes of IL-27 level. Note: The abscissa indicated the time nodes, and the ordinate indicated the level, pg/ml. The IL-27 levels of the CG before treatment, at 4 weeks, 8 weeks, and 12 weeks of treatment were (105.86 ± 47.33), (83.74 ± 24.08), (76.55 ± 34.88), and (70.22 ± 30.43). The IL-27 levels of the SG before treatment, at 4 weeks, 8 weeks, and 12 weeks of treatment were (104.98 ± 46.74), (68.57 ± 21.26), (64.71 ± 29.69), and (59.87 ± 25.57). ^∗^indicates the obvious difference in the IL-27 level at 4 weeks of treatment between both groups (*t* = 3.558, *P* < 0.001).

**Table 1:** Comparison of general data (*n* = 60).

Observation indexes	ACS group	SA group	Non-CHD group	*P*
Age (years old)	67.52 ± 6.11	67.84 ± 6.23	67.61 ± 6.10	>0.05
BMI (kg/m^2^)	23.75 ± 3.08	23.88 ± 3.05	23.83 ± 3.06	>0.05
Heart rate (times/min)	74.71 ± 14.12	75.06 ± 14.02	74.85 ± 12.07	>0.05
Systolic blood pressure (mmHg)	110.52 ± 12.31	110.46 ± 12.28	110.50 ± 12.25	>0.05
Diastolic blood pressure (mmHg)	78.94 ± 10.03	79.07 ± 10.02	79.03 ± 10.01	>0.05
Gender				>0.05
Male	34 (56.67)	32 (53.33)	33 (55)	
Female	26 (43.33)	28 (46.67)	27 (45)	
Smoking	25 (41.67)	23 (38.33)	24 (40)	>0.05
Drinking	27 (45)	28 (46.67)	27 (45)	>0.05
Education degree				
Below high school degree	38 (63.33)	35 (58.33)	36 (60)	>0.05
Senior high school degree	8 (13.33)	10 (16.67)	11 (18.33)	>0.05
Junior high school degree and above	14 (23.33)	15 (25)	13 (21.67)	>0.05
Underlying diseases				
Diabetes	3 (5)	4 (6.67)	3 (5)	>0.05
Hypertension	12 (20)	11 (18.33)	11 (18.33)	>0.05
Hyperlipidemia	3 (5)	5 (8.33)	4 (6.67)	>0.05
Chronic renal insufficiency	1 (1.67)	1 (1.67)	1 (1.67)	>0.05

**Table 2:** Changes of serum RBP4, hs-CRP, and IL-27 levels.

Group	RBP4 (mg/L)	Hs-CRP (mg/L)	IL-27 (mg/L)
ACS group	36.87 ± 13.04	5.83 ± 2.71	116.57 ± 43.55
SA group	24.34 ± 8.05^∗^	4.35 ± 1.02^∗^	83.42 ± 27.19^∗^
Non-CHD group	9.32 ± 3.71^∗^#	1.88 ± 0.44^∗^#	24.55 ± 5.16^∗^#

^∗^indicates *P* < 0.05 compared with the ACS group, and # indicates *P* < 0.05 compared with the SA group.

**Table 3:** Correlation between Gensini score and serum RBP4, hs-CRP, and IL-27 levels.

		RBP4	Hs-CRP	IL-27
Gensini score	Related coefficient	0.797^∗∗^	0.817^∗∗^	0.809^∗∗^
	Sig.	0.000	0.000	0.000

^∗∗^indicates that the correlation was significant at a confidence (bilateral) of 0.01.

## Data Availability

The data are available on reasonable request from the corresponding author.
